The article "A Network Pharmacology to Explore the Mechanism of Calculus Bovis in the Treatment of Ischemic Stroke" was retracted in 2024. Reasons: suspected computer-generated content; unreliable results or conclusions; concerns about the data; concerns about the results or conclusions.

# A Network Pharmacology to Explore the Mechanism of *Calculus Bovis* in the Treatment of Ischemic Stroke

**DOI:** 10.1155/2021/6611018

**Published:** 2021-03-10

**Authors:** Fangchen Liu, Ling Li, Jian Chen, Ying Wu, Yongbing Cao, Ping Zhong

**Affiliations:** ^1^Department of Neurology, Shanghai TCM-Integrated Hospital, Shanghai University of Traditional Chinese Medicine, Shanghai 200082, China; ^2^Shanghai University of Traditional Chinese Medicine, Shanghai 201203, China; ^3^Institute of Vascular Disease, Shanghai TCM-Integrated Hospital, Shanghai University of Traditional Chinese Medicine, Shanghai 200082, China; ^4^Department of Neurology, Shidong Hospital of Yangpu District, Shanghai 200090, China

## Abstract

**Background:**

*Calculus Bovis* is a valuable Chinese medicine, which is widely used in the clinical treatment of ischemic stroke. The present study is aimed at investigating its target and the mechanism involved in ischemic stroke treatment by network pharmacology.

**Methods:**

Effective compounds of *Calculus Bovis* were collected using methods of network pharmacology and using the Bioinformatics Analysis Tool for Molecular Mechanism of Traditional Chinese Medicine (BATMAN-TCM) and the Traditional Chinese Medicine Systems Pharmacology Database and Analysis Platform (TCMSP). Potential compound targets were searched in the TCMSP and SwissTargetPrediction databases. Ischemic stroke-related disease targets were searched in the Drugbank, DisGeNet, OMIM, and TTD databases. These two types of targets were uploaded to the STRING database, and a network of their interaction (PPI) was built with its characteristics calculated, aiming to reveal a number of key targets. Hub genes were selected using a plug-in of the Cytoscape software, and Gene Ontology (GO) biological processes and pathway enrichment analyses of Kyoto Encyclopedia of Genes and Genomes (KEGG) were conducted using the clusterProfiler package of R language.

**Results:**

Among 12 compounds, deoxycorticosterone, methyl cholate, and biliverdin were potentially effective components. A total of 344 *Calculus Bovis* compound targets and 590 ischemic stroke targets were found with 92 overlapping targets, including hub genes such as TP53, AKT, PIK2CA, MAPK3, MMP9, and MMP2. Biological functions of *Calculus Bovis* are associated with protein hydrolyzation, phosphorylation of serine/threonine residues of protein substrates, peptide bond hydrolyzation of peptides and proteins, hydrolyzation of intracellular second messengers, antioxidation and reduction, RNA transcription, and other biological processes.

**Conclusion:**

*Calculus Bovis* may play a role in ischemic stroke by activating PI3K-AKT and MAPK signaling pathways, which are involved in regulating inflammatory response, cell apoptosis, and proliferation.

The article "A Network Pharmacology to Explore the Mechanism of Calculus Bovis in the Treatment of Ischemic Stroke" was retracted in 2024. Reasons: suspected computer-generated content; unreliable results or conclusions; concerns about the data; concerns about the results or conclusions.

## 1. Introduction

Stroke is an acute cerebrovascular disease with typical clinical manifestations of sudden weakness in one side of the face, arms, or legs; sudden faintness; and unconsciousness. Ischemic stroke, the most common form of stroke, accounts for 70-80% of the total number of cases among stroke patients [1]. In China, deaths due to cerebrovascular diseases accounted for more than 20% of the total deaths in 2018 [2]. The rehabilitation of patients with ischemic stroke is often ineffective which brings a heavy burden to society and families. Currently, tissue-type plasminogen activator (tPA) is the only approved treatment for acute ischemic stroke [3–5]. However, its clinical application is greatly limited due to the narrow treatment time window, high bleeding risk, and many contraindications [6]. In China, stroke has been managed with herbs or other Chinese methods for thousands of years. Chinese herbal medicine are now widely accepted as the main complementary treatment in East Asia, North America, and Europe because of their good therapeutic effect, low toxicity, and low cost [7–9].

*Calculus Bovis*, one of the most commonly used Chinese herbs for stroke, has been used for over 2,000 years in China. It was first described in “Shen Nong Ben Cao Jing” as a medication with a bitter taste and cooling nature [10]. And it has been applied in conditions like loss of consciousness due to stroke, epilepsy, mania, and other mental disorders. It was shown that *Calculus Bovis* protects the brain through its anti-inflammatory, antiapoptosis [11], antilipid peroxidation [12], and antioxidative stress effects [13]. It is well known that herbs have multiple ingredients targeting multiple sites and multiple pathways [14, 15]. Currently, *Calculus Bovis* and its formulas are widely used to treat ischemic stroke, but the mechanisms underlying its therapeutic effect have not been studied intensively.

Network pharmacology for Chinese herbs is developed to decipher interactions between herbs and diseases at a system level by analysing the network between herbs, compounds, targets, diseases, and genes [16–19]. In the present study, our aim is to reveal the underlying mechanisms of *Calculus Bovis* in managing ischemic stroke by network pharmacology methods, which will lay the foundation for future pharmacological and clinical studies on ischemic stroke. The protocol of our experimental procedures is shown in Figure 1.

## 2. Materials and Methods

### 2.1. Data Acquisition

#### 2.1.1. Prediction of Compounds of *Calculus Bovis* and Their Targets

Compounds of *Calculus Bovis* were collected from the herbal platform TCMSP and BATMAN-TCM. The TCMSP (https://tcmspw.com/tcmsp.php) is a systems pharmacology platform for herbs providing information about compounds and their targets [20]. The BATMAN-TCM (http://bionet.ncpsb.org/batman-tcm/) is an online bioinformatics analysis tool comprised of functions like target prediction for herbs and target analysis [21]. When “NIU HUANG (*Calculus Bovis*)” was typed in the “Cluster name,” “Score cutoff” value was set at 20, and “Adjusted *p* value” was set at 0.05, compounds of *Calculus Bovis* and their targets would be displayed. In addition, potential targets could be searched in the TCMSP and SwissTargetPrediction (http://www.swisstargetprediction.ch/) databases [22] to further confirm the targets of compounds derived from *Calculus Bovis*. Names of target proteins were translated into gene names in the UniProt (http://www.uniprot.org/) database. If there was overlap in their target genes, the duplicates were deleted. Similarly, when the gene names of the protein targets were not found in the Uniprot database, they were deleted. SMILES IDs of compounds contained in *Calculus Bovis* were searched in the PubChem (https://pubchem.ncbi.nlm.nih.gov/) database, and their targets were predicted using SwissTargetPrediction after setting “*Homo sapiens*.” After collecting targets from the TCMSP, BATMAN-TCM, and SwissTargetPrediction databases, the duplicates were deleted.

The article "A Network Pharmacology to Explore the Mechanism of Calculus Bovis in the Treatment of Ischemic Stroke" was retracted in 2024. Reasons: suspected computer-generated content; unreliable results or conclusions; concerns about the data; concerns about the results or conclusions.

#### 2.1.2. Prediction of Pharmacodynamics

In pharmacological studies, absorption, distribution, metabolism, and excretion (ADME) are key indices for identifying specific drugs [23]. Herein, 2 key parameters related to ADME, namely, oral bioavailability (OB) and drug-like activities (DL), were analyzed to explore potential bioactive compounds in *Calculus Bovis*. Based on the content of known compounds, OB and DL were set at ≥15% and ≥0.1, respectively. It has been reported that ergosterol (MOL000298; OB: 14.29%: DL: 0.72) is an indispensable compound of *Calculus Bovis* [24, 25] and was included in the present study. All compounds included in the present study were supported by the literature.

#### 2.1.3. Collection of Disease Targets of Ischemic Stroke

Key words such as “ischemic stroke,” “cerebral ischemic stroke,” and “brain ischemia” were used, and “*Homo sapiens*” was selected for species. They were searched in the Drugbank [26], DisGeNet [27], OMIM [28], and TTD databases [29], and duplicate genes were deleted.

#### 2.1.4. Venny Plotting

Both compound targets and disease targets were uploaded to the website of Venny 2.1.0 (https://bioinfogp.cnb.csic.es/tools/venny/); overlapping genes were the potential targets of bioactive compounds, and they interact with the body in ischemic stroke.

The article "A Network Pharmacology to Explore the Mechanism of Calculus Bovis in the Treatment of Ischemic Stroke" was retracted in 2024. Reasons: suspected computer-generated content; unreliable results or conclusions; concerns about the data; concerns about the results or conclusions.

#### 2.1.5. Protein-Protein Interaction (PPI)

The STRING (https://string-db.org) database has collected a large number of well-known or predicted protein-protein interaction results [30]. Overlapping genes from Venny plots were uploaded to the database and “*Homo sapiens*” was selected for species, high confidence (0.700) was set for the minimum required interaction score, and irrelevant targets were concealed. As a result, a network map showing interactions between individual targets was rendered.

### 2.2. Network Construction and Hub Gene Selection

Network analysis facilitates interpretation of relationships between herbs, compounds, diseases, and genes. In the present study, two networks were constructed using Cytoscape 3.7.0 (https://cytoscape.org/) [31]: (1) a network of *Calculus Bovis* compounds and compound targets and (2) a PPI network of *Calculus Bovis* compound targets and a PPI network of *Calculus Bovis* treating ischemic stroke targets after connecting *Calculus Bovis* compound targets and disease targets. Topographical analysis for networks was completed using the NetworkAnalyzer tool in Cytoscape. Overlapping genes, also named Hub genes, were selected from the PPI networks using the cytoHubba plug-in in Cytoscape and 3 algorithms were used in the calculations. The latter included degree of freedom, Maximum Neighborhood Component (MNC), and Maximal Clique Centrality (MCC).

### 2.3. Gene Functions and Pathway Enrichment Analysis

Gene Ontology (GO) enrichment analysis and Kyoto Encyclopedia of Genes and Genomes (KEGG) pathway analysis were conducted using the clusterProfiler package of R (R 4.0.2 for Windows) to identify biological processes and pathways with systemic involvement. Biological processes and pathways with a significant difference were selected, and their numbers of enrichment as well their as *p* values were ranked. The top 20 results from the GO enrichment and KEGG pathway enrichment analyses were presented. Visualization of these pathways with a *p* value < 0.05 was completed using the R software package.

## 3. Results and Analysis

A total of 12 bioactive compounds were found after ADME screening, and all of them have been verified in other studies.

### 3.1. *Calculus Bovis* Compound-Target Network

A total of 344 targets were found by 12 bioactive compounds of *Calculus Bovis*. Details of these ingredients are listed in Table 1, and the map of the compound-target network is shown in Figure 2. Circles represent compounds of *Calculus Bovis*, and triangles represent the targets; their colors are darkened as their degrees of freedom increased. There were 362 nodes and 706 edges with a network density of 0.011 and a network diameter of 5. Details of these parameters are listed in Table 2.

The article "A Network Pharmacology to Explore the Mechanism of Calculus Bovis in the Treatment of Ischemic Stroke" was retracted in 2024. Reasons: suspected computer-generated content; unreliable results or conclusions; concerns about the data; concerns about the results or conclusions.

### 3.2. Disease Targets of Ischemic Stroke

Using key words listed in Section 2.1.3, 74 disease targets were found in the Drugbank database, 313 were found in the DisGeNet database after screening for values above the average, 322 were found in the OMIM database, and 10 were found in the TTD database. A total of 590 targets were found after deleting gene duplicates.

### 3.3. Prediction of *Calculus Bovis* Targets in Ischemic Stroke

After entering compound targets and disease targets to Venny 2.1.0 in the form of gene names, 92 overlapping genes were found (see Figure 3). These genes were the shared targets of the bioactive compounds and disease targets in ischemic stroke.

### 3.4. Construction of PPI Networks

#### 3.4.1. The PPI Network of *Calculus Bovis* Targets

PPI networks have been widely used in studying protein-protein interactions in different diseases. To construct the PPI network of *Calculus Bovis* targets, 12 compounds were connected with 344 targets in the TCMSP and the SwissTargetPrediction databases, and they were imported into the STRING database (species: *Homo sapiens*; minimum required interaction score: high confidence (0.700)), and the PPI network was visualized after reconstructing it with Cytoscape (version 3.7.0). As shown in Figure 4, colors darkened as the degree of freedom increased. This PPI network contained 322 nodes and 2195 edges with a diameter of 8 and an average number of neighbors of 13.634. It showed that TP53 (degree = 82), AKT1 (degree = 67), MAPK1 (degree = 67), PIK3CA (degree = 63), SRC (degree = 58), MAPK3 (degree = 56), VEGFA (degree = 52), HSP90AA1 (degree = 48), JUN (degree = 46), EGFR (degree = 46), MAPK8 (degree = 45), TNF (degree = 40), and CASP3 (degree = 40) were the key nodes of this PPI network.

#### 3.4.2. The PPI Network of *Calculus Bovis*-Ischemic Stroke Targets and Hub Genes

To explore the potential therapeutic mechanisms of *Calculus Bovis* in managing ischemic stroke, 92 shared targets by *Calculus Bovis* compounds and ischemic stroke were connected and imported into the STRING database as shown in Figure 5(a). The PPI network of *Calculus Bovis*-ischemic stroke targets were constructed by visualizing the results using Cytoscape (Figure 5(b)). This PPI network had 83 nodes and 403 edges with a network diameter of 6 and an average number of neighbors of 9.711. The top 10 targets with the highest degree of freedom were TP53 (degree = 33), AKT1 (degree = 30), MAPK1 (degree = 29), VEGFA (degree = 27), TNF (degree = 25), PIK3CA (degree = 25), MAPK3 (degree = 24), MMP9 (degree = 22), PTGS2 (degree = 22), and IL-1B (degree = 20). A total of 6 Hub genes were found using 3 algorithms: degree of freedom, Maximum Neighborhood Component (MNC), and Maximal Clique Centrality (MCC) (Figure 5(c)). These genes were TP53, AKT1, PIK3CA, MAPK3, MMP9, and MMP2. Their network of interactions is shown in Figure 5(d). In addition, TP53, AKT1, MAPK1, VEGFA, PIK3CA, and MAPK3 were among the top 10 candidates ranked by degree of freedom.

The article "A Network Pharmacology to Explore the Mechanism of Calculus Bovis in the Treatment of Ischemic Stroke" was retracted in 2024. Reasons: suspected computer-generated content; unreliable results or conclusions; concerns about the data; concerns about the results or conclusions.

### 3.5. GO Enrichment Analysis

To further investigate the underlying mechanism of *Calculus Bovis* in managing ischemic stroke, 344 targets and 92 shared targets were collected for GO enrichment analysis.

#### 3.5.1. GO Enrichment Analysis for *Calculus Bovis* Targets

Twenty results were selected based on their *p* values and their numbers of enrichment. They were primarily involved in ion channel activity (GO:0005216), channel activity (GO:0015267), passive transmembrane transporter activity (GO:0022803), gated channel activity (GO:0022836), cation channel activity (GO:0005261), metal ion transmembrane transporter activity (GO:0046873), neurotransmitter receptor activity (GO:0030594), ligand-gated ion channel activity (GO:0015276), ligand-gated channel activity (GO:0022834), postsynaptic neurotransmitter receptor activity (GO:0098960), extracellular ligand-gated ion channel activity (GO:0005230), neurotransmitter receptor activity involved in regulation of postsynaptic membrane potential (GO:0099529), transmitter-gated ion channel activity (GO:0022824), transmitter-gated channel activity (GO:0022835), and steroid dehydrogenase activity (GO:0016229). Details are listed in Table 3. Results are presented using a bubble plot and a column chart using the R package.

*(1) Bubble Plot*. In the bubble plot, letters on the left are GO names, numbers on the bottom are the proportions of genes, sizes of circles indicate the numbers of enriched genes, and colors reflect *p* values. The redder the colors are, the more enriched the genes are, and the smaller the *p* values are (Figure 6).

*(2) Column Chart*. In the column chart, letters on the left are GO names, numbers on the bottom are the numbers of genes enriched on GO, and *p* reflects significance of enrichment. The redder the colors are, the more enriched the genes are, and the smaller the *p* values are (Figure 7).

#### 3.5.2. GO Enrichment Analysis of Shared Targets of *Calculus Bovi*s and Ischemic Stroke

GO enrichment analysis was performed against the 92 shared targets. The top 20 were selected based on their *p* values and numbers of enrichment, including endopeptidase activity (GO:0004175); protein serine/threonine kinase activity (GO:0004674); metallopeptidase activity (GO:0008237); phosphoric diester hydrolase activity (GO:0008081); heme binding (GO:0020037); tetrapyrrole binding (GO:0046906); oxidoreductase activity, acting on paired donors, with incorporation or reduction of molecular oxygen (GO:0016705); serine-type peptidase activity (GO:0008236); serine hydrolase activity (GO:0017171); carboxylic acid binding (GO:0031406); organic acid binding (GO:0043177); metalloendopeptidase activity (GO:0004222); RNA polymerase II transcription factor binding (GO:0001085); monocarboxylic acid binding (GO:0033293); and fatty acid binding (GO:0005504) (see Table 4). Results were visualized as a bubble plot (Figure 8) and a column chart (Figure 9) using the R package.

The article "A Network Pharmacology to Explore the Mechanism of Calculus Bovis in the Treatment of Ischemic Stroke" was retracted in 2024. Reasons: suspected computer-generated content; unreliable results or conclusions; concerns about the data; concerns about the results or conclusions.

### 3.6. KEGG Pathway Enrichment Analysis

KEGG pathway enrichment analysis was performed for 344 *Calculus Bovis* targets and 92 shared targets.

#### 3.6.1. KEGG Pathway Enrichment Analysis for *Calculus Bovis* Targets

Eighteen results were selected based on their *p* values and their numbers of enrichment. They were mainly involved in neuroactive ligand-receptor interaction (hsa04080), Alzheimer disease (hsa05010), calcium signaling pathway (hsa04020), nicotine addiction (hsa05033), steroid hormone biosynthesis (hsa00140), GABAergic synapse (hsa04727), morphine addiction (hsa05032), cholinergic synapse (hsa04725), retrograde endocannabinoid signaling (hsa04723), and cellular senescence (hsa04218) (see Table 5).

*(1) Bubble Plot*. In the bubble plot, letters on the left are KEGG names, numbers on the bottom are the proportions of genes, sizes of circles indicate the numbers of enriched genes, and colors reflect *p* values. The redder the colors are, the more enriched the genes are, and the smaller the *p* values are (Figure 10).

*(2) Column Chart*. In the column chart, letters on the left are KEGG names, numbers on the bottom are the numbers of genes enriched on KEGG, columns represent genes enriched on KEGG, and *p* reflects significance of enrichment. The redder the colors are, the more enriched the genes are, and the smaller the *p* values are (Figure 11).

#### 3.6.2. KEGG Pathway Enrichment Analysis for Shared Targets

KEGG pathway enrichment analysis was performed on 92 shared targets, and 145 pathways were found. The top 20 candidates were selected based on their *p* values and numbers of enrichment, and they were involved in the PI3K-AKT signaling pathway (hsa04151), human papillomavirus infection (hsa05165), Kaposi sarcoma-associated herpesvirus infection (hsa05167), human cytomegalovirus infection (hsa05163), microRNAs in cancer (hsa05206), fluid shear stress and atherosclerosis (hsa05418), proteoglycans in cancer (hsa05205), AGE-RAGE signaling pathway in diabetic complications (hsa04933), cAMP signaling pathway (hsa04024), prostate cancer (hsa05215), TNF signaling pathway (hsa04668), platelet activation (hsa04611), EGFR tyrosine kinase inhibitor resistance (hsa01521), small cell lung cancer (hsa05222), and endocrine resistance (hsa01522) (Table 6). Results were visualized as a bubble plot (Figure 12) and a column chart (Figure 13) using the R package.

The article "A Network Pharmacology to Explore the Mechanism of Calculus Bovis in the Treatment of Ischemic Stroke" was retracted in 2024. Reasons: suspected computer-generated content; unreliable results or conclusions; concerns about the data; concerns about the results or conclusions.

## 4. Discussion

Network pharmacology was used in this study to investigate *Calculus Bovis* itself and its potential mechanism for the treatment of ischemic stroke through compound target network construction, PPI network analysis, GO enrichment analysis, and KEGG pathway analysis.

Network analysis of compound targets showed that deoxycorticosterone (MOL008846), methyl cholate (MOL008838), and biliverdin (MOL008834) had the most connections with these targets, suggesting that these 3 compounds might be the key compounds of *Calculus Bovis*.

Deoxycorticosterone is a type of steroid hormone possessing activities of the mineralocorticoid and serves as the precursor of aldosterone. It is involved in water and salt metabolism, playing an important role in electrolyte balance and in the volume of body fluid [32]. It has been reported that deoxycorticosterone and its derivatives—neurosteroids transformed in the fetal brain—protect the central nervous system. Inhibiting the production of neurosteroids increases basal cell death [33]. Neuroactive steroid hormones are involved in the regulation of diverse physiological functions, such as cell differentiation, neuroprotection, memory reinforcement, and amelioration of anxiety and pressure [34]. Methyl cholate is the methyl ester form of cholic acid, inhibiting the synthesis of cholesterol [35]. It has been reported that methyl cholate suppresses the growth of certain Gram-positive and Gram-negative bacteria [36] and has a good anti-inflammatory effect [37]. Biliverdin is a type of bile pigment, an oxidized product of heme. Emerging evidence has shown that biliverdin is an endogenous antioxidant facilitating the restoration of the tissue oxidation-reduction environment [38]. In the middle cerebral artery occlusion (MCAO) model, it significantly decreased the infarct area and the production of peroxides in the cortex [39]. These indicate that biliverdin plays a pivotal role in mitigating ischemic brain injury through its antioxidative stress effect. In addition, a single target was regulated by multiple compounds as shown in our network. Protein-tyrosine phosphatase 1B (PTPN1) was subject to the regulation of deoxycorticosterone, oleanolic acid, ergosterol, ursolic acid, biliverdin, bilirubin, methyl cholate, methyl desoxycholate, taurodeoxychloic acid, and others. PTPs are involved in regulating differentiation and survival of neurons and have also been reported to be a new target of antiplatelet therapy [40]. PTPN1 is a negative regulator of the leptin and insulin signaling pathways, and PTP1B knockout mice are exempt from obesity and diabetes, both of which are risk factors of ischemic stroke [41].

The article "A Network Pharmacology to Explore the Mechanism of Calculus Bovis in the Treatment of Ischemic Stroke" was retracted in 2024. Reasons: suspected computer-generated content; unreliable results or conclusions; concerns about the data; concerns about the results or conclusions.

Similarly, other targets like 11-beta-hydroxysteroid dehydrogenase 1 (HSD11B1), dual-specificity phosphatase Cdc25A (CDC25A), cytochrome P450 19A1 (CYP19A1), progesterone receptor (PGR), and androgen receptor (AR) were also regulated by two or more compounds. The present study revealed not only relationships between *Calculus Bovis* compounds and their targets but also the potential pharmacological effects of *Calculus Bovis*, which reflects the multicompound and multitarget theory of modern drugs.

Furthermore, the PPI network demonstrated information not only about protein homology and coexpression but also about protein-protein interactions. Our PPI analysis showed that *Calculus Bovis* influences ischemic stroke through its impact on a complex biological network, including TP53, AKT1, MAPK1, VEGFA, TNF, PIK3CA, MAPK3, MMP9, PTGS2, and IL1B. Hub gene screening revealed that TP53, AKT1, PIK3CA, MAPK3, MMP9, and MMP2 were essential in this process. The above potential targets for the action of *Calculus Bovis* in the treatment of ischemic stroke are our first discoveries.

TP53, cellular tumor antigen p53, is a tumor suppressing gene. It promotes cell apoptosis, increases gene stability, and suppresses tumorigenesis [42]. It has been reported that methylation of the TP53 promoter was increased in ischemic stroke, and this increase was associated with the thickness of the intima of the carotid artery, degree of atherosclerosis of the carotid artery, and levels of homocysteine in the peripheral blood [43]. More evidence showed that TP53 induced glycolysis, and apoptosis regulator (TIGAR) suppressed glycolysis, increased pentose-phosphate pathway flux, and maintained the function of mitochondria. As a result, it protected the brain from ischemic injury [44]. The Tp53 Arg/Arg genotype has been considered a genetic marker for predicting poor prognosis after ischemic stroke [45]. AKT1 (serine/threonine-protein kinase AKT) codes for the serine/threonine-protein kinase which regulates apoptosis proteins and transcription factors. It is the key player in regulating cell survival, growth, apoptosis, and proliferation in the presence of growth factors and external stimuli, especially brain ischemia and reperfusion injury. AKT1 gene variance is closely related to metabolic syndrome, a risk factor of stroke [46].

The article "A Network Pharmacology to Explore the Mechanism of Calculus Bovis in the Treatment of Ischemic Stroke" was retracted in 2024. Reasons: suspected computer-generated content; unreliable results or conclusions; concerns about the data; concerns about the results or conclusions.

AKT/PKB was involved in brain ischemia, and its activity was related to the extent of ischemic injury. Activation of AKT was the key factor in determining survival of neurons after ischemic injury [47]. PIK3CA codes for the p110 subunit of the phosphatidylinositol 3-kinases (PI3Ks), and its mutations decrease cell apoptosis and increase the activity of downstream PI3Ks. It is known that activation of PI3K/AKT promotes repair of neural injury due to ischemic stroke [48, 49] and angiogenesis in the hypoxic environment in vitro [50]. Consequently, it protects the rat brain from inflammation resulting from ischemia-reperfusion injury [51]. Activation of the TrkB/PI3K/AKT pathway also increases activation of Nrf2 and its translocation to the nucleus, which plays a pivotal role in protecting the central nervous system from oxidative stress [52].

MAPK (mitogen-activated protein kinase) is involved in reaction to physiological and pathological stimuli, such as cytokines, neurotransmitters, hypoxia, and hypoglycemia [53]. MAPK3 (MAP kinase ERK1) and MAPK1 (MAP kinase ERK2) form ERK1/2, a subfamily of MAPK. They play important roles in cell proliferation, differentiation, migration, invasion, apoptosis, and other biological processes. In the H_2_O_2_ induced PC12 cell injury model, activation of the AKT and ERK1/2 pathways leads to an antioxidation effect [54]. Levels of ERK1 and ERK2 were increased after ischemic stroke onset. In vitro research further revealed that activation of ERK1/2 increased neuronal apoptosis, indicating that they are important targets for ischemic stroke treatment [55].

GO and KEGG pathway enrichment analyses for *Calculus Bovis* targets showed that *Calculus Bovis* was closely related to ion channel activity, neurotransmitter receptor activity, and other physiological functions. Pathway enrichment analysis demonstrated its involvement in a number of pathways in the central nervous system, calcium-related signaling, and so on. These were consistent with the analgesic and antiepilepsy effects of *Calculus Bovis* and its clinical application in these fields, which lays the theoretical foundation for managing ischemic stroke using *Calculus Bovis*.

GO enrichment and KEGG pathway analyses against the shared 92 targets showed that *Calculus Bovis* was closely related to hydrolyzation of proteins, phosphorylation of serine/threonine residues of protein substrates, peptide bond hydrolyzation of peptides and proteins, hydrolyzation of second intracellular messengers, antioxidation and reduction, RNA transcription, and other biological processes. Among them, 15 (16.3%) were related to endopeptidase activities of the matrix metalloproteinase (MMPs) family (MMP1, MMP2, MMP3, MMP8, MMP9, MMP10, and MMP12) and the cysteine-containing aspartate-specific peptidase family (CASP1, CASP2, and CASP3). MMPs are a type of highly conserved proteinase in nature, belonging to the family of zinc-dependent endopeptidases. They are capable of degrading extracellular matrix, growth factors, cytokines, and cell adhesion molecules. They are indispensable in ECM and tissue remodeling, angiogenesis, immune reactions, inflammation, cell migration, proliferation, cell apoptosis, and other physiological and pathological processes [56]. Their mRNAs were dramatically increased in the cortex of the mouse ischemia model in which thrombus was induced [57]. Decreasing levels of MMPs significantly ameliorated transgression of neutrophils, which resulted in neuroprotection against ischemic stroke [58]. Targeted inhibition of the PI3K/AKT/MMP-9 signaling pathway suppressed tumor invasion and metastasis [59], but this has not been tested in neuronal cells. Caspases are closely related to apoptosis of eukaryocytes and regulation of cell proliferation as well as differentiation. Caspase 3 is the most important and indispensable one in the cascade of cell apoptosis. In brain ischemia, levels of CASP3 mRNA and protein were increased, and its activity was significantly reversed by a CASP3 inhibitor, preventing the hydrolyzation of poly(ADP-ribose) polymerase. Consequently, apoptosis was suppressed and neurological functions improved [60]. Neuroinflammation is a key pathological process, in which CASP1-activated inflammasomes play an essential role. It has been reported that CASP1 was increased in the mouse brain after cerebral ischemia, which was suppressed by a CASP1 inhibitor through decreasing the activation of microglial cells, protecting the brain from ischemic injury. These indicate that CASP1 is a potential drug target for ischemic stroke management [61]. Both in vitro and in vivo experiments have shown that activation of the PI3K/AKT pathway increases the phosphorylation of Bad and decreases the level of caspase-3, through which apoptosis is suppressed [62].

The article "A Network Pharmacology to Explore the Mechanism of Calculus Bovis in the Treatment of Ischemic Stroke" was retracted in 2024. Reasons: suspected computer-generated content; unreliable results or conclusions; concerns about the data; concerns about the results or conclusions.

Another 12 genes (13.0%) are related to activities of protein serine/threonine kinases, consistent with the findings of the PI3K-AKT signaling pathway (24 enriched genes, 27.2%) in the KEGG pathway analysis. AKT is also named serine/threonine kinase, whose activation is key for neuronal survival [63]. It is known that phosphorylated AKT was decreased in the infarct area after ischemia-reperfusion injury and increased in the penumbra after reperfusion. An inhibitor of PI3K decreased the level of phosphorylated AKT and increased the infarct area, indicating that PI3K/AKT is involved in the pathogenesis of brain ischemia and activation of AKT increases neuronal survival [64]. Among them, MAPK3 (ERK1) is not only a Hub gene involved in regulating the activity of protein serine/threonine kinases as shown by GO analysis but is also enriched in the PI3K-AKT signaling pathway. These suggest that MAPK3 is an important component of this network. Therefore, *Calculus Bovis* might protect the brain from ischemic stroke through its anti-inflammatory and antiapoptosis effects which are accomplished by interacting with the abovementioned key genes and pathways.

However, there are some limitations in this study. Access to databases of Chinese herbal medicines and disease targets is relatively limited, and there may be some data selection bias. Meanwhile, due to the fact that this study was based on data analysis, the conclusion needs to be confirmed by further research.

## 5. Conclusion

Bioactive compounds, potential targets, and underlying mechanisms of *Calculus Bovis* were examined using network pharmacology methods. KEGG pathway analysis showed that the PI3K/AKT and the MAPK signaling pathways were the key targets for ischemic stroke treatment. The effect of *Calculus Bovis* was achieved through directly or indirectly regulating the above targets and pathways. Our results confirmed that *Calculus Bovis* was a multicompound and multitarget drug with a multisystem character in the treatment of ischemic stroke, which laid the theoretical foundation for the development of drugs and therapeutic methods based on the results of *Calculus Bovis* in the future.

## Figures and Tables

**Figure 1:** The schematic map of the present study.

**Figure 2:** *Calculus Bovis* compound-target network. Note: circles represent compounds, triangles represent targets, and their colors darken as their degrees of freedom increase.

**Figure 3:** Venny diagram of *Calculus Bovis* targets and ischemic stroke disease targets. CB: *Calculus Bovis* target; IS: ischemic stroke disease target.

**Figure 4:** Protein-protein interaction (PPI) network of *Calculus Bovis* compound targets. Darkness of colors and sizes of circles represent the degree of freedom as the scale indicates.

**Figure 5:** The PPI network of *Calculus Bovis* compound targets against ischemic stroke (IS): (a) the original PPI data generated from the STRING database showing detailed interactions of the targets; (b) the PPI network constructed using Cytoscape (version 3.7.0); (c) the top 15 genes were calculated from the PPI network by the degree of freedom, MNC, and MCC, and the overlapping genes were then screened by Venn diagrams; (d) the PPI network of hub genes.

The article "A Network Pharmacology to Explore the Mechanism of Calculus Bovis in the Treatment of Ischemic Stroke" was retracted in 2024. Reasons: suspected computer-generated content; unreliable results or conclusions; concerns about the data; concerns about the results or conclusions.

**Figure 6:** Bubble plot of GO enrichment analysis of *Calculus Bovis* targets. Bubble plot: letters on the left are GO names, numbers on the bottom are the proportions of genes, sizes of the circles indicate the numbers of enriched genes, and colors reflect *p* values. The redder the colors are, the more enriched the genes are, and the smaller the *p* values are.

**Figure 7:** Column chart of GO functional enrichment analysis of *Calculus Bovis* targets. Column chart: letters on the left are GO names, numbers on the bottom are the numbers of genes enriched on GO, and *p* reflects the significance of enrichment. The redder the colors are, the more enriched the genes are, and the smaller the *p* values are.

**Figure 8:** Bubble plot of GO enrichment analysis of shared targets by *Calculus Bovis* and ischemic stroke.

**Figure 9:** Column chart of GO enrichment analysis of shared targets by *Calculus Bovis* and ischemic stroke.

**Figure 10:** Bubble plot of KEGG pathway enrichment analysis of *Calculus Bovis* targets. Bubble plot: letters on the left are KEGG names, numbers on the bottom are the proportions of genes, sizes of the circles indicate the numbers of enriched genes, and colors reflect *p* values. The redder the colors are, the more enriched the genes are, and the smaller the *p* values are.

**Figure 11:** Column chart of KEGG pathway enrichment analysis of *Calculus Bovis* targets. Column chart: letters on the left are KEGG names, numbers on the bottom are the numbers of genes enriched on KEGG, columns represent genes enriched on KEGG, and *p* reflects the significance of enrichment. The redder the colors are, the more enriched the genes are, and the smaller the *p* values are.

**Figure 12:** Bubble plot of KEGG pathway enrichment analysis of shared targets.

**Figure 13:** Column chart of KEGG pathway enrichment analysis of shared targets.

**Table 1:** Active ingredients of *Calculus Bovis*.

Mol ID	Mol name	2D structure	OB (%)	DL
MOL000263	Oleanolic acid		29.02	0.76
MOL000298	Ergosterol		14.29	0.72
MOL000511	Ursolic acid		16.77	0.75
MOL008834	Bilicerdin		23.79	0.75
MOL008835	3-[2-[[3-(2-Carboxyethyl)-4-methyl-5-[(E)-(4-methyl-5-oxo-3-vinyl-2-pyrrolylidene)methyl]-1H-pyrrol-2-yl]methyl]-4-methyl-5-[(Z)-(3-methyl-5-oxo-4-vinyl-2-pyrrolylidene)methyl]-1H-pyrrol-3-yl]propanoic acid		16.53	0.75
MOL008838	Methyl (4R)-4-[(3R,5S,7S,8R,9S,10S,12S,13R,14S,17R)-3,7,12-trihydroxy-10,13-dimethyl-2,3,4,5,6,7,8,9,11,12,14,15,16,17-tetradecahydro-1H-cyclopenta[a]phenanthren-17-yl]pentanoate		32.32	0.76
MOL008839	Methyl desoxycholate		34.63	0.73
MOL008840	2-[(3alpha,12alpha-Dihydroxy-24-oxo-5beta-cholan-24-yl)amino]ethanesulfonic acid		15.92	0.87
MOL008843	Cherianoine		27.32	0.12
MOL008846	ZINC01280365		46.38	0.49
MOL000953	CLR		37.87	0.68
MOL009807	CHD		22.17	0.72

Abbreviations: OB = oral bioavailability; DL = drug likeness; Mol = molecular.

The article "A Network Pharmacology to Explore the Mechanism of Calculus Bovis in the Treatment of Ischemic Stroke" was retracted in 2024. Reasons: suspected computer-generated content; unreliable results or conclusions; concerns about the data; concerns about the results or conclusions.

**Table 2:** *Calculus Bovis* compound-candidate target network parameters.

Network parameters	Values
Number of nodes	362
Network density	0.011
Network diameter	5
Network heterogeneity	3.212
Average number of neighbors	3.901
Characteristic path length	3.236
Shortest paths	130682 (100%)
Network centralization	0.304

**Table 3:** GO enrichment analysis results of *Calculus Bovis* targets.

No.	ID	Description	Count	*p* value
1	GO:0005216	Ion channel activity	14	1.15918 × 10^−10^
2	GO:0015267	Channel activity	14	3.57104 × 10^−10^
3	GO:0022803	Passive transmembrane transporter activity	14	3.67058 × 10^−10^
4	GO:0022836	Gated channel activity	13	7.88226 × 10^−11^
5	GO:0005261	Cation channel activity	11	1.25701 × 10^−8^
6	GO:0046873	Metal ion transmembrane transporter activity	11	1.85161 × 10^−7^
7	GO:0030594	Neurotransmitter receptor activity	9	1.68357 × 10^−10^
8	GO:0015276	Ligand-gated ion channel activity	8	1.76915 × 10^−8^
9	GO:0022834	Ligand-gated channel activity	8	1.76915 × 10^−8^
10	GO:0098960	Postsynaptic neurotransmitter receptor activity	7	3.22861 × 10^−9^
11	GO:0005230	Extracellular ligand-gated ion channel activity	6	1.78299 × 10^−7^
12	GO:0099529	Neurotransmitter receptor activity involved in regulation of postsynaptic membrane potential	5	6.54501 × 10^−7^
13	GO:0022824	Transmitter-gated ion channel activity	5	1.78703 × 10^−6^
14	GO:0022835	Transmitter-gated channel activity	5	1.78703 × 10^−6^
15	GO:0016229	Steroid dehydrogenase activity	4	5.40 × 10^−6^
16	GO:0016628	Oxidoreductase activity, acting on the CH-CH group of donors, NAD or NADP as acceptor	4	1.58 × 10^−6^
17	GO:1904315	Transmitter-gated ion channel activity involved in regulation of postsynaptic membrane potential	4	1.78589 × 10^−5^
18	GO:0022851	GABA-gated chloride ion channel activity	3	9.83 × 10^−6^
19	GO:0042166	Acetylcholine binding	3	2.32 × 10^−5^
20	GO:0015271	Outward rectifier potassium channel activity	3	1.56 × 10^−5^

**Table 4:** GO enrichment analysis results of shared targets by *Calculus Bovis* and ischemic stroke.

No.	ID	Description	Count	*p* value
1	GO:0004175	Endopeptidase activity	15	5.14505 × 10^−9^
2	GO:0004674	Protein serine/threonine kinase activity	12	2.81896 × 10^−6^
3	GO:0008237	Metallopeptidase activity	9	4.20451 × 10^−7^
4	GO:0008081	Phosphoric diester hydrolase activity	8	3.02315 × 10^−8^
5	GO:0020037	Heme binding	8	5.05803 × 10^−7^
6	GO:0046906	Tetrapyrrole binding	8	8.71647 × 10^−7^
7	GO:0016705	Oxidoreductase activity, acting on paired donors, with incorporation or reduction of molecular oxygen	8	1.74788 × 10^−6^
8	GO:0008236	Serine-type peptidase activity	8	4.78249 × 10^−6^
9	GO:0017171	Serine hydrolase activity	8	5.61466 × 10^−6^
10	GO:0031406	Carboxylic acid binding	8	7.36664 × 10^−6^
11	GO:0043177	Organic acid binding	8	1.14448 × 10^−5^
12	GO:0004222	Metalloendopeptidase activity	7	1.07557 × 10^−6^
13	GO:0001085	RNA polymerase II transcription factor binding	7	1.62174 × 10^−5^
14	GO:0033293	Monocarboxylic acid binding	6	9.84665 × 10^−7^
15	GO:0005504	Fatty acid binding	5	8.40369 × 10^−7^
16	GO:0043560	Insulin receptor substrate binding	4	2.19487 × 10^−7^
17	GO:0036041	Long-chain fatty acid binding	4	6.57868 × 10^−7^
18	GO:0004114	3′,5′-Cyclic-nucleotide phosphodiesterase activity	4	1.27273 × 10^−5^
19	GO:0004112	Cyclic-nucleotide phosphodiesterase activity	4	1.47051 × 10^−5^
20	GO:0016303	1-Phosphatidylinositol-3-kinase activity	3	1.58908 × 10^−5^

The article "A Network Pharmacology to Explore the Mechanism of Calculus Bovis in the Treatment of Ischemic Stroke" was retracted in 2024. Reasons: suspected computer-generated content; unreliable results or conclusions; concerns about the data; concerns about the results or conclusions.

**Table 5:** KEGG pathway enrichment analysis results of *Calculus Bovis* targets.

No.	ID	Description	Count	*p* value
1	hsa04080	Neuroactive ligand-receptor interaction	14	1.03 × 10^−8^
2	hsa05010	Alzheimer disease	9	4.14 × 10^−6^
3	hsa04020	Calcium signaling pathway	6	3.4 × 10^−5^
4	hsa05033	Nicotine addiction	5	2.08104 × 10^−4^
5	hsa00140	Steroid hormone biosynthesis	5	2.31001 × 10^−4^
6	hsa04727	GABAergic synapse	5	3.04528 × 10^−4^
7	hsa05032	Morphine addiction	5	3.73161 × 10^−4^
8	hsa04725	Cholinergic synapse	5	6.29559 × 10^−4^
9	hsa04723	Retrograde endocannabinoid signaling	5	1.033601 × 10^−3^
10	hsa04218	Cellular senescence	5	1.40748 × 10^−3^
11	hsa04330	Notch signaling pathway	4	1.594499 × 10^−3^
12	hsa04115	p53 signaling pathway	4	2.068787 × 10^−3^
13	hsa05204	Chemical carcinogenesis	4	2.107734 × 10^−3^
14	hsa04540	Gap junction	4	2.532292 × 10^−3^
15	hsa04970	Salivary secretion	4	2.652055 × 10^−3^
16	hsa04914	Progesterone-mediated oocyte maturation	4	3.294802 × 10^−3^
17	hsa05030	Cocaine addiction	3	3.367718 × 10^−3^
18	hsa04340	Hedgehog signaling pathway	3	3.567181 × 10^−3^

**Table 6:** KEGG pathway enrichment analysis for shared targets.

No.	ID	Description	Count	*p* value
1	hsa04151	PI3K-AKT signaling pathway	24	2.12708 × 10^−13^
2	hsa05165	Human papillomavirus infection	20	2.45479 × 10^−10^
3	hsa05167	Kaposi sarcoma-associated herpesvirus infection	19	1.3448 × 10^−13^
4	hsa05163	Human cytomegalovirus infection	18	2.23341 × 10^−11^
5	hsa05206	MicroRNAs in cancer	18	4.23388 × 10^−9^
6	hsa05418	Fluid shear stress and atherosclerosis	17	8.25476 × 10^−14^
7	hsa05205	Proteoglycans in cancer	17	4.88669 × 10^−11^
8	hsa04933	AGE-RAGE signaling pathway in diabetic complications	16	6.21323 × 10^−15^
9	hsa04024	cAMP signaling pathway	16	1.04013 × 10^−9^
10	hsa05215	Prostate cancer	14	1.54571 × 10^−12^
11	hsa04668	TNF signaling pathway	14	1.16611 × 10^−11^
12	hsa04611	Platelet activation	13	6.34665 × 10^−10^
13	hsa01521	EGFR tyrosine kinase inhibitor resistance	12	3.67514 × 10^−11^
14	hsa05222	Small cell lung cancer	12	2.32309 × 10^−10^
15	hsa01522	Endocrine resistance	12	4.93414 × 10^−10^
16	hsa04919	Thyroid hormone signaling pathway	12	5.80768 × 10^−9^
17	hsa05212	Pancreatic cancer	11	4.36655 × 10^−10^
18	hsa05210	Colorectal cancer	11	1.70773 × 10^−9^
19	hsa04657	IL-17 signaling pathway	11	4.49095 × 10^−9^
20	hsa05220	Chronic myeloid leukemia	10	7.44115 × 10^−9^

The article "A Network Pharmacology to Explore the Mechanism of Calculus Bovis in the Treatment of Ischemic Stroke" was retracted in 2024. Reasons: suspected computer-generated content; unreliable results or conclusions; concerns about the data; concerns about the results or conclusions.

## Data Availability

The data used to support the findings of this study are included within the article.

## Supplementary Materials

Supplementary Materials Supplementary 1. Table S1: all ingredients of *Calculus Bovis*. Supplementary 2. Table S2: targets of active ingredients of *Calculus Bovis*.
